RETRACTED

# Awareness of Medical Students toward Circadian Rhythm and Sleep Disorder Based on Biomedical Diagnosis

**DOI:** 10.1155/2022/8645183

**Published:** 2022-08-18

**Authors:** Asma Alanazi, Haifa Alhawas, Munirah Aldossari, Dana Almutairi, Dana Almatroudi, Afnan Alenazi, Leen Almadhi, Maram Albalawi

**Affiliations:** ^1^Department of Basic Medical Sciences, College of Medicine, King Saud bin Abdulaziz University for Health Sciences (KSAU-HS), Riyadh, Saudi Arabia; ^2^King Abdullah International Medical Research Center, Riyadh, Saudi Arabia; ^3^Department of Biostatistics and Bioinformatics, King Abdullah International Medical Research Center, Riyadh, Saudi Arabia

## Abstract

**Background:**

Sleep disorders affect an individual's mental and physical health and vice versa. Sleep medicine is underrecognized as a specialty; therefore, many sleep disorders go undiagnosed. This study is aimed at assessing the knowledge of medical students toward circadian neuroscience and sleep disorder based on biomedical diagnosis.

**Methods:**

This cross-sectional study was conducted in both male and female medical colleges from the third to the sixth year. A self-administered structured questionnaire consisting of sociodemographic data and the Assessment of Sleep Knowledge in Medical Education (ASKME) survey assessed the students' general knowledge and attitude towards sleep disorder and sleep medicine. Chi-square/Fisher exact tests were used to analyse the participants' knowledge level toward specific sociodemographic data. Also, for two-level continuous variables, the Wilcoxon two-sample test was used.

**Results:**

The total number of participants was 296, with 154 female and 142 male participants. The prevalence of inadequate knowledge was considerable with 96.62% of students, compared to adequate knowledge with only 3.38%. The students' attitude to sleep medicine was negative 14.53% and positive among 85.47%. We found that gender was significantly associated with attitude with a *p* value = 0.0057. The specific interest in sleep medicine had a significant association with knowledge and attitude, *p* value of 0.0522 and 0.0059, respectively.

**Conclusion:**

This study concluded that medical students possess inadequate knowledge regarding sleep medicine, yet they have a positive attitude towards it.

## 1. Introduction

Sleep affects an individual's mental health and psychological state due to its close connection to mental health [1]. As sleep can affect one's mental health, having mental health problems could lead to sleep disorders [1]. Sleep disorders are defined as a disturbance in an individual's sleep pattern [2]. It can be caused by various environmental conditions and factors [2]. Delayed sleep phase disorder, shift work sleep disorder, restless leg syndrome, insomnia, and sleep apnea are common sleep disorders [2].

RETRACTED

Moreover, sleep disorders are prevalent among Saudi medical students, especially female students, according to a study done by Abdulghani et al. [3]. The need for sleep medicine, a medical specialty that focuses on sleep-related problems, is anticipated to increase significantly due to the increased prevalence of sleep disorders in the Saudi population [4]. Both sleep disorders and sleep medicine are underrecognized by healthcare workers and public workers [5]. Sleep medicine specialties' underrecognition could be because it is a relatively new specialty in the medical profession [5]. The latest International Classification of Sleep Disorders (ICSD) approved that more than seventy disorders were divided into seven major categories [6]. Although there are accurate diagnostic instruments and efficient therapies for many sleep disorders, sleep testing and treatments are still unavailable [7]. There are many sleep disorders and inadequate numbers of sleep health professionals in parts of the world [7]. According to a study conducted in Saudi Arabia in 2007, there are limited studies investigating the prevalence of sleep disorders, although there are widespread sleep disorders among the Saudi population [8]. A survey revealed that sleep medicine in Saudi Arabia is underdeveloped compared to developed countries, and there are two main problems facing the progress of this specialty [8]. One of these obstacles includes an insufficient number of sleep-medicine experts and a lack of insurance coverage and funding [8]. Both health workers and general health practitioners do not consider sleep medicine an independent specialty [5].

Moreover, most people in Saudi Arabia do not have adequate knowledge about sleep medicine and sleep disorders. Since sleep medicine is a relatively new specialty, many people do not acknowledge its existence—people in the healthcare profession, especially medical students, lack awareness of sleep medicine as a specialty. According to a study conducted at Qassim University, medical students appeared to have limited knowledge about sleep medicine, but they showed a positive attitude towards it [9]. A study was done to assess the knowledge of sleep medicine among medical students in Riyadh and found that over 80% of the students rated their knowledge of sleep medicine to be below average [10]. In addition, it claimed that it is an obstacle that sleep medicine is considered a low priority in the medical school curriculum [10]. Early detection of specific sleeping disorders depends on the knowledge of the Primary Healthcare (PHC) physician in KSA. However, insufficient education on sleep medicine during medical school and residency training leads to inadequate knowledge in physicians, which would compromise the quality of patient care [5].

RETRACTED

Moreover, since the physicians are uninformed about sleep medicine, patients with sleeping disorders go undiagnosed, which may lead to further complications [11]. Furthermore, Saudi PHC physicians do not fully understand sleep medicine as a specialty. According to Saleem et al.'s study, 25.7% of participant physicians admit that they would not take sleep medicine history from their patients as an essential part of their history-taking practice [12]. Moreover, 39.2% deem sleep disturbances a lifestyle problem rather than a medical condition [12]. Also, only 63% of physicians realize that obstructive sleep apnea (OSA) increases the risk of motor vehicle accidents, as mentioned in the BaHammams study [13].

According to several studies, OSA is prevalent among PHC physicians' clinic patients [13–16]. However, OSA and other sleep disorders commonly go undiagnosed because sleep medicine is underdeveloped as a specialty; hence, there is a lack of specialists, especially in KSA [5, 8]. It is impractical to expect a limited amount of sleep medicine specialists to diagnose all the sleep disorders. Alternatively, educational interventions have proven to help raise the awareness and diagnosis of sleep disorders among PHC physicians [17]. Consequently, the primary purpose of this study was to assess the knowledge and attitude regarding sleep medicine among medical students at King Saud bin Abdulaziz University for Health Sciences (KSAU-HS), Riyadh branch, using a cross-sectional study.

## 2. Methods

Based on an online survey, a cross-sectional study was conducted in KSAU-HS, Riyadh branch, regarding the knowledge and attitude of medical students towards sleep medicine as a specialty. The study population included medical students. The inclusion criteria were male and female medical students from the third year to the sixth year. The exclusion criteria were graduated students as well as those whose data were incomplete. The Raosoft sample size calculator was used to calculate the sample size with a population size of 1200 students, a 95% confidence interval, a margin of error of 5%, and the response distribution was 50% of medical students with adequate knowledge. Therefore, the sample size became 292.

The data collection was through a self-administered questionnaire consisting of three parts: each part consists of closed-end questions. The three parts were, namely, sociodemographic data, knowledge about sleep and sleep disorder, and attitude toward sleep medicine. The first part of the questionnaire is about the student's sociodemographic characteristics (age, year of study, gender, GPA, preferred specialty, specific interest in sleep medicine, and students' perspective on the importance of sleep medicine). The second part assesses the students' knowledge about sleep medicine using the Assessment of Sleep Knowledge in Medical Education (ASKME) survey [18]. Experts developed and validated the questionnaire using a pilot study to find reliability. The questionnaire contains a 30-question survey in which the outcome variables were (a) questions on students' knowledge of basic sleep principles, (b) circadian sleep/wake control, (c) normal sleep architecture, (d) common sleep disorders, and (e) the effect of drugs and alcohol on sleep. Each question had four choices: one correct answer, two wrong answers, and an “I do not know” choice. The correct answer was coded as one, while all the other answers were coded as zero.

RETRACTED

The minimum score was 0, and the maximum score was 30 after summing up the score of thirty questions. Participants were classified into two categories by applying the cutoff points of 18/30 (60% of the total score). If the score range was from 0 to 17 points, we classified them as having inadequate knowledge; on the other hand, if the score range was from 18 to 30 points, the student's knowledge was categorized as adequate knowledge. The third part assesses the participants' attitudes toward sleep and sleep disorder using a questionnaire containing ten questions adapted from the ASKME survey [18]. The response to the attitude questions was a 5-point Likert scale (from strongly agree = 5 to strongly disagree = 1). The total score ranged from 10 to 50. Participants who scored 30 (60% of the total score) or more were categorized as having a positive attitude. In contrast, the participants whose scores were less than 30 were categorized as having a negative attitude.

## 3. Data Analysis

All data analyses were performed using the Statistical Analysis System (SAS) Version 9.4 software. Descriptive statistics for all qualitative variables will be presented as numbers and percentages, while the mean ± standard deviation for all quantitative variables will be presented. Chi-square/Fisher exact tests were used to analyse the participants' knowledge level with the sociodemographic profile (gender, GPA, year of study, and specific interest). Additionally, the Wilcoxon two-sample test was used for two-level continuous variables. The *p* value < 0.05 will be considered statistically significant for all tests applied with a 95% confidence interval.

RETRACTED

The study proposal was approved by the King Abdullah International Medical Research Center (KAIMRC), registered at the National Committee of Bio & Med. Ethics (NCBE) (Registration No. SP21R\168\04). Consent was taken through the questionnaire, and no personal information was taken from the participants. In addition, the participants were given no compensation or benefit in any form. Only the research team had access to all the data, as all the data was kept classified throughout the entire study.

## 4. Results

The questionnaire was distributed randomly among the third-, fourth-, fifth-, and sixth-year medical students, and there were 296 responses. The sociodemographic characteristics of the students who participated in this study are listed in Table 1. The students' ages were classified from less than 25 to more than 25; most of the participants, 280 (94.5%), were under 25 years old, with a slight inclination towards the female respondents being 154 (52%). The fourth-year medical student had the highest responses compared to the other students. Moreover, most of the participants, 272 (91.89%), had a 4.1 or higher (GPA). According to their preferred area of specialization, many students preferred medicine as a specialty 169 (57.09%). Most of the participants are not interested in sleep medicine, 240 (81.08%); despite that, many students believe sleep medicine is important.

Table 2 represents the result of the ASKME questionnaire, which indicates the number of correct responses. The questions that had the highest correct response rate were “when does the body increase the secretion of melatonin,” “how much time do newborn infants spend sleeping per 24 hours,” and “what can increase the incidence of sleepwalking in children” with 77.36%, 76.69%, and 61.49% of students answering it correctly, respectively. The question that had the least correct responses was “what is recommended in patients with difficulty in initiating sleep” with 17 (5.74%) students.

The general attitude of the medical students in this study is presented in Figure 1. Most of the students disagreed with every statement, especially statements 1 and 7. However, most of the students agreed with statement 8, with 94 (31.76%) strongly agreeing and 125 (42.23%) agreeing. In addition, statement 4 had mixed responses in which 28.04% responses were neutral, and the choices “agree” and “disagree” had approximate percentages 24.32% and 22.64%, respectively.

The characteristics of the students' knowledge and attitude toward sleep medicine in Table 3 show that the mean knowledge score was 10.09 (±4.15) out of 30. In this study, the prevalence of inadequate knowledge was considerable with 286 (96.62%) students, compared to adequate knowledge with 10 (3.38%) students. The mean attitude score was 35.56 (±5.61) out of 50. Moreover, only 43 (14.53%) participants had a negative attitude towards sleep medicine, whereas 253 (85.47%) participants had a positive attitude toward it.

RETRACTED

Table 4 shows the comparison between sociodemographic data of participants and their knowledge and attitude scores. There is statistical significance in the positive attitude of females compared to males with a *p* value = 0.0057, although their knowledge scores are not statistically significant. Using the Wilcoxon test, the mean score of students' knowledge and attitude with a specific interest is higher and statistically significant with a *p* value = 0.0522 for the knowledge and a *p* value of 0.0059 for the attitude than those who do not have a specific interest.

## 5. Discussion

The main goal of this study was to assess the knowledge and attitude of medical students at King Saud bin Abdulaziz University for Health Sciences toward circadian neuroscience and sleep disorder based on biomedical diagnosis. The final analysis found that the students' knowledge was poor 286 (96.62%). In another study conducted in 2020 at King Abdulaziz University in Jeddah by Alghamdi et al., the ASKME questionnaire was used [19]. They classified the results into two categories: low scores (<60%) and high scores (>60%) [19]. A total of 568 medical students participated, out of which the mean score was 9.89 (±4.89) and 97.7% had low scores [19]. Additionally, they found no statistically significant difference between both genders' knowledge scores as the findings in this study [19]. Another local study done at Qassim University by Alrebdi et al. had 116 medical students [9]. While using the ASKME questionnaire, they found that 94.8% of the participants had poor knowledge with positive attitude among the students, which was consistent with the results of this study [9]. In a study from Egypt, they had 726 participants complete the survey, of which there were 573 sixth-year medical students [20, 21]. Their results indicated poor knowledge among medical students [22]. Furthermore, there was a statistically significant difference in the knowledge scores of participants' gender and the knowledge scores, which conflicts with our findings [23, 24].

## 6. Conclusion

The medical students in the KSAU-HS Riyadh branch have poor knowledge toward sleep disorder and sleep medicine, indicating a need for sleep medicine to be added to the medical curriculum of KSAU-HS. Also, the students' positive attitude towards sleep medicine demonstrates that they are willing to learn about it. To acquire proper knowledge among medical students, we recommend that the professors be educated about sleep medicine and its importance in the medical field. In our study, there is a significant association between attitude and gender. Also, there is a significant association between knowledge and attitude with a specific interest in sleep medicine. However, our study did not find any association between GPA or year of study and sleep medicine.

RETRACTED

The study is a cross-sectional study with its limitation of not being the perfect representation of the population over time. Moreover, there might be a misinterpretation of questions. Finally, there is a lack of introspective ability among the participants as the survey is self-reported, affecting the results.

Due to the lack of studies in this area, it is recommended to increase the sample population in future studies and to include more colleges and medical specialties in Saudi Arabia.

## Figures and Tables

**Figure 1:** General attitude of the students toward sleep medicine.

**Table 1:** Sociodemographic characteristics of participants (*n* = 296).

Study variables	*N* (%)
Gender	
(i) Female	154 (52)
(ii) Male	142 (47.97)

Age	
(i) Less than 25	280 (94.5)
(ii) More than 25	16 (5.41)

Year of study	
(i) 3^rd^ year	70 (23.65)
(ii) 4^th^ year	93 (31.42)
(iii) 5^th^ year	65 (21.96)
(iv) 6^th^ year	68 (22.97)

GPA	
(i) 2.4-4.0	24 (8.11)
(ii) 4.1-5.0	272 (91.89)

Preferred specialty	
(i) Medicine	169 (57.09)
(ii) Surgery	88 (29.73)
(iii) Others	39 (13.18)

Specific interest in sleep medicine	
(i) Yes	56 (18.92)
(ii) No	240 (81.08)

Importance of sleep medicine	
(i) Absolutely not important	7 (2.36)
(ii) Not important	10 (3.38)
(iii) Average	76 (25.68)
(iv) Important	104 (35.14)
(v) Very important	99 (33.45)

**Table 2:** General knowledge toward circadian and sleep disorder based on biomedical diagnosis (*n* = 296).

Knowledge questions	Correct answers *N* (%)
(Q1) When does the need for sleep decrease in a person?	144 (48.65)
(Q2) When does the body increase its secretion of melatonin?	229 (77.36)
(Q3) When does dream sleep or rapid eye movement sleep (REM) occur?	168 (56.76)
(Q4) How does a person make up for his loss of sleep during the work week?	179 (60.47)
(Q5) How much time do newborn infants spend sleeping per 24 hours?	227 (76.69)
(Q6) What is the prevalence of insomnia between older men and women?	35 (11.82)
(Q7) What should we do to a young (preadolescent) child who regularly has trouble getting to sleep at night?	59 (19.93)
(Q8) What is the typical age of symptom onset for narcolepsy?	43 (14.53)
(Q9) When does the ability to sleep increase?	86 (29.05)
(Q10) When is the slow-wave sleep more prominent?	52 (17.57)
(Q11) When does the amount of slow-wave sleep increase?	35 (11.82)
(Q12) Episodes of sleepwalking tend to occur which third of the night?	77 (26.01)
(Q13) When do episodes of REM sleep tend to lengthen?	124 (41.89)
(Q14) During REM sleep, what happens to periodic limb movements?	74 (25)
(Q15) In children, inadequate sleep can exacerbate which of the following?	48 (16.22)
(Q16) With alcoholics in recovery, how long of alcohol abstention does it take to normalize their sleep?	24 (8.11)
(Q17) What is recommended in patients with difficulty in initiating sleep?	17 (5.74)
(Q18) What is often an indicator in the treatment of primary snoring or mild obstructive sleep apnea?	116 (39.19)
(Q19) What enhanced slow-wave sleep?	63 (21.28)
(Q20) What drug could cause chronic bedwetting in children?	120 (40.54)
(Q21) Nightmare are more common within?	49 (16.55)
(Q22) Heart rate, respiration, and blood pressure are more variable during?	100 (33.78)
(Q23) Do antihypertensive drugs cause sleep difficulties as side effects?	50 (16.89)
(Q24) What is true regarding early morning awakening in the elderly?	99 (33.45)
(Q25) What is correct regarding the benefit from alcohol?	159 (53.72)
(Q26) What statement is correct?	158 (53.38)
(Q27) Episode of sleepwalking commonly occurs at which stage?	49 (16.55)
(Q28) Who is at higher risk of developing symptoms of sleep apnea?	146 (49.32)
(Q29) What can increase the incidence of sleepwalking in children?	182 (61.49)
(Q30) What is the most symptom that correlates with narcolepsy?	75 (25.34)

RETRACTED

**Table 3:** Knowledge and attitude.

Predictor variable	*N* (%)
Level of knowledge	
(i) Adequate	10 (3.38)
(ii) Inadequate	286 (96.62)

Attitude	
(i) Positive	253 (85.47)
(ii) Negative	43 (14.53)

Knowledge score (mean ± SD)	10.09 ± 4.15

Attitude total score (mean ± SD)	35.56 ± 5.61

**Table 4:** Comparison between the sociodemographic data.

*N* = 296	Knowledge		Attitude	
	Adequate *N* (%)	Inadequate *N* (%)	Positive *N* (%)	Negative *N* (%)
Gender				
Female	6 (3.9)	148 (96.1)	140 (90.91)	14 (9.09)
Male	4 (2.82)	138 (97.18)	113 (79.58)	98 (20.48)
*p* value	0.7518		0.0057^∗^	
GPA				
4.1-5	9 (3.31)	263 (96.69)	234 (86.03)	38 (13.97)
2.4-4	1 (4.17)	23 (95.83)	19 (79.17)	5 (20.83)
*p* value	0.5765		0.3651	
Year of study				
3^rd^ year	1 (1.43)	69 (98.57)	58 (82.86)	12 (17.14)
4^th^ year	2 (2.15)	91 (97.85)	77 (82.8)	16 (17.2)
5^th^ year	4 (6.15)	61 (93.85)	59 (90.77)	6 (9.23)
6^th^ year	3 (4.41)	65 (95.59)	59 (86.76)	9 (13.24)
*p* value	0.4059		0.4785	
Specific interest				
Yes	3 (5.36)	53 (94.64)	49 (87.5)	7 (12.5)
No	7 (2.92)	233 (97.08)	204 (85)	36 (15)
*p* value	0.0522^∗^		0.0059^∗^	

^∗^Significant at *p* ≤ 0.05.

## Data Availability

The data used to support the findings of this study are included within the article.
